# The Risk and Clinical Treatment of Hypertensive Diseases in Pregnant Women

This article has been retracted.

**DOI:** 10.1155/2022/8480106

**Published:** 2022-09-05

**Authors:** Jie Xu, Xin Yu, Zhimin Wang

**Affiliations:** ^1^Department of Obstetrics, Laiyang Central Hospital of Yantai, Laiyang, 265200 Shandong, China; ^2^Department of Obstetrics, Ji'nan Maternal and Child Health Hospital, Jinan, 250000 Shandong, China

## Abstract

Hypertensive disorders of pregnancy are a group of pregnancy-related diseases characterized by the coexistence of pregnancy and elevated blood pressure, which seriously endanger the health of mothers and infants, and are one of the main causes of maternal and perinatal deaths. The purpose of this paper is to investigate the clinical analysis of vitamin E and astragalus in the adjuvant treatment of hypertensive disorders in pregnancy and to describe the learning model. This paper puts forward the problem of clinical treatment, which is established on the basis of adjuvant therapy, then narrates around the clinical characteristics of gestational hypertension, and designs and analyzes the experimental design and analysis of adjuvant therapy with vitamin E and astragalus. The experimental results showed that the delivery methods of the three groups of patients were compared *P* < 0.05. Compared with the traditional Chinese medicine control group and the vitamin E control group, there were more vaginal births in the experimental group, 36 patients in total. It shows that astragalus and vitamin E can alleviate the disease in different aspects and can effectively intervene in gestational hypertension.

## 1. Introduction

Hypertensive disorder of pregnancy is a pregnancy-related disorder that seriously affects the health of mothers and babies. The incidence rate in China and abroad is 9.4%-10.4% and 7%-12%, respectively, which is the disease with the highest incidence and the most difficult treatment in obstetrics. Despite doctors' increased understanding of the disease and advanced medical methods, current treatments remain unsatisfactory. Therefore, researchers at home and abroad have begun to pay attention to the early diagnosis and timely treatment of the disease.

The influencing factors of gestational hypertension are still unclear. Therefore, in-depth research on the incidence of gestational hypertension, maternal and infant prognosis, and related factors can help to prevent and reduce its occurrence and is of great significance to protect the health of pregnant women and fetuses. The purpose of this study is to study the efficacy, safety, and possible mechanism of vitamin E and astragalus in the treatment process, to find the best time for treatment, and to provide a new approach and theoretical basis for the treatment of hypertensive disorders in pregnancy.

The innovations of this paper are the following: (1) This paper combines gestational hypertension with vitamin E and astragalus and introduces the theory and related methods of the learning model in detail. The support vector machine model, logistic regression model, and hidden Markov model are mainly introduced. (2) Clinical analysis of using vitamin E and astragalus is adjuvant therapy in the face of gestational hypertension. By evaluating the experimental results and comparing the effects of vitamin E and astragalus on various indicators of pregnant women, it is concluded that astragalus and vitamin E play an intervention role in gestational hypertension.

## 2. Related Work

Hypertensive disorders of pregnancy are diseases specific to pregnancy, and hypertensive disorders of pregnancy remain one of the leading causes of maternal and fetal morbidity and mortality in humans, both in developed and developing countries. Pedersen et al. investigated the effects of ambient air pollution and road traffic noise on gestational hypertensive disorders in a Danish national birth cohort of 72745 cases (1997-2002). The findings suggest that road traffic may increase the risk of preeclampsia and hypertensive disorders in pregnancy through exposure to ambient air pollution and noise, although the associations with these two exposures are generally not independent of each other. However, they did not give specific recommendations [1]. Facco et al. aimed to test a major hypothesis that sleep-disordered breathing during pregnancy is associated with an increased incidence of preeclampsia. The experimental results showed that sleep-disordered breathing was independently associated with preeclampsia, pregnancy-induced hypertension, and GDM. However, they did not take into account other influencing factors [2]. Alvarez-Alvarez et al. experimented with the hypothesis that pregnancy-induced hypertension (PIH) causes maternal and infant damage but may also be the start of future metabolic and vascular disease. Women with a history of preeclampsia/eclampsia had twice the risk of stroke, a higher frequency of cardiac arrhythmias, and hospitalizations for heart failure. They also observed a 10-fold increased risk of developing long-term chronic kidney disease. The relative risk of cardiovascular death was 2.1-fold higher compared with the group without PIH problems, although the risk of preterm birth associated with gestational hypertension or preexisting hypertension was 4- to 7-fold higher. However, they have insufficient contrast [3]. Azliana et al. conducted a retrospective cross-sectional study from January 1, 2015, to December 31, 2015, evaluating a total of 30 placentas. Studies have shown that the increased number of syncytial nodules in the placenta of HDP patients is a consistent histological finding. The expression of VEGF was significantly increased in placental syncytiotrophoblasts in the hypertensive group, which can be used as a biomarker of hypertension. However, his experimental data is less [4]. Kyozuka et al. study the relationship between preconception sodium (Na) intake and HDP development in normotensive women. The study design was derived from the Japan Environment and Children Study (JECS) database, which identified 85152 normotensive Japanese women enrolled in JECS between January 2011 and March 2014. It was concluded that in normotensive Japanese women, both lower and higher preconception sodium intake increased the risk of HDP with SGA. This finding may suggest new recommendations for preconception Na intake to prevent HDP. However, there are certain subjective thoughts in their conclusion [5]. Li et al. investigate the effects of prepregnancy body mass index (BMI) and gestational weight gain (GWG) on childhood overweight and obesity and explore early risk factors for obesity in preschool children. However, their data is unclear [6]. The aim of Acharya et al. was to compare the perinatal outcomes of neonates delivered by hypertensive and normal mothers. Their hospital-based comparative study was conducted at the Nipargun Medical College Teaching Hospital, Khoharpur, from December 2014 to December 2015. Fifty mothers who met the inclusion criteria and their fetal outcomes (stillbirths and neonates) were selected for the study, and 50 normal normotensive healthy mothers and their neonatal or fetal outcomes were selected as the control group. Experiments show that compared with normal pregnancies, pregnancy with hypertension is characterized by an increased incidence of preterm birth and low birth weight infants. However, they did not specify the specific impact [7]. Sun et al. used stepwise logistic regression and the lasso method to compare the model effects of two range selections and selected the PlGF model with a good prediction effect and suitable gestational age for final prediction. The final model of the lasso method in his study is more effective by comprehensive comparison. According to clinical needs and model effect, the best HDP prediction model with PlGF parameters in the second trimester (15-26 weeks) was finally selected. However, their performance needs to be improved [8].

## 3. Learning Model Approach for Clinical Treatment

### 3.1. Learning Model

#### 3.1.1. Support Vector Machine Model

Support vector machines were first proposed in the 1980s and are mainly used to deal with data classification problems, especially binary classification problems; such problems can be Boolean such as true or false or numerical such as 1 or -1. SVM can not only be applied to low-dimensional space but also shows excellent performance in high-dimensional space, and the computational efficiency is also very high. In addition, it also has good generalization ability, is suitable for small sample classification space, and only needs a few samples to train to obtain a classifier with good performance and high efficiency. Therefore, SVM is widely used in industry and is a very attractive and promising development direction [9, 10]. As shown in Figure 1, assuming that there are two types of data sets, we hope to find a decision surface that can separate the two types of data. The decision surface here refers to a straight line between two types of data. Both sides of the decision surface can be divided into positive and negative classes, which are represented by 1 and -1.

When mapping sample points to a higher-dimensional space, such a problem sometimes occurs. After mapping to a higher-dimensional space, the classification problem cannot be solved, so it must be mapped to a higher-dimensional space to solve it. And so, it may have to calculate to a particularly high number of dimensions, which leads to high-dimensional disaster. In order to alleviate this problem and reduce the amount of computation, the concept of kernel function is introduced. The kernel function transforms the linearly inseparable samples in the low-dimensional space to make them linearly separable in the high-dimensional space. In layman's terms, when a problem is not linearly separable, SVM's approach is to perform calculations in a lower-dimensional space and then select an appropriate kernel function to map the data to a high-dimensional space. By making the samples linearly separable by this mapping, SVM can also be combined with different algorithms. Therefore, different forms of kernel-based methods can be used to solve different problems.

Using SVM to separate the two types of data by interval is to find a hyperplane that can maximize the distance. If not found, map the data to a higher dimensional space. For example, for the left plot in Figure 2, the data is linearly inseparable in two-dimensional space; that is, there is no way to find a straight line to separate the data into two categories. So, by matching the data to 3D space, it is easy to find the segmentation hyperplane and classify the data [11].

SVM does not arbitrarily choose a straight line between two data sets; in fact, there are many straight lines that can achieve data partitioning. In order to maximize the distance between them, SVM needs to find the one that maximizes the distance between two different points among these lines. As shown in Figure 3, the larger the classification interval, the more accurate the judgment of new sample points, and the situation that the interval is small and easy to misclassify is avoided as much as possible. Therefore, SVM requires the classification interval to be as large as possible, that is, to find the straight line with the largest interval, and if it is mapped to the high-dimensional space, it is to find the hyperplane with the largest interval.

Taking the two-class problem as an example, for a given sample set (*m*_*a*_, *n*_*a*_), *a* = 1, 2, ⋯, *i*, *m*_*a*_ is the *a*th sample and *n*_*a*_ is the label corresponding to the *i*th sample; assuming that the problem is linearly separable, *n*_*a*_ ∈ {+1, −1}, then the hyperplane formula is

(1) $$\begin{array}{c} w\cdot m+j=0, \end{array}$$

where *m* is the input vector, *w* is the weight vector, and *j* is the bias.

In order for the model to correctly classify all samples and ensure the maximum classification interval, the following conditions need to be met:

(2) $$\begin{array}{c} \left\{\begin{array}{c} w\cdot m_{a}+j\geq +1,\;n_{a}=+1,\\ w\cdot m_{a}+j\leq -1,\;n_{a}=-1. \end{array}\right. \end{array}$$

That is,

(3) $$\begin{array}{c} n_{a}\left(w\cdot m_{a}+j\right)\geq 1,\;a=1,2,\cdots ,i. \end{array}$$

Under the condition of obeying the above constraints, the maximization of the classification interval 2/‖*w*‖ is achieved, which is transformed into the minimization function under the constraints:

(4) $$\begin{array}{c} \varphi \left(w\right)=\frac{1}{2}{\left\|w\right\|}^{2}=\frac{1}{2}\left(w\cdot w\right). \end{array}$$

#### 3.1.2. Logistic Regression Model

Logistic regression is a common classification method that trains a logistic function to make predictions on new samples, such as spam filtering. The popularity of email is convenient for everyone, but it also brings some troubles. Spam content affects normal communication and brings bad user experience to users. It is necessary to use a certain strategy to classify emails into normal emails and spam emails. The simplest idea is to set a threshold for classification based on the continuous-valued results predicted by linear regression [12]. In fact, this method of setting thresholds can be used to solve simple cases. For example, when diagnosing a disease, the tumor size of many samples is known to determine whether a new sample is a malignant tumor. First, a linear regression model *h*_*ϑ*_(*w*) is established, and then, a threshold is set, such as 0.5. When *h*_*ϑ*_(*w*) ≥ 0.5, the point is judged to be a malignant tumor; otherwise, when *h*_*ϑ*_(*w*) < 0.5, the point is judged to be a benign tumor. However, the actual example is much more complicated, and there are often some interfering data that cannot be linearly separable. At this time, logistic regression is introduced. The function of the logistic regression model is defined as

(5) $$\begin{array}{c} h_{\vartheta }\left(w\right)=g\left(s\right). \end{array}$$

In the formula, *s* = *ϑ*^*T*^*w*, *w* is the feature vector, function *g* is the sigmoid function, and its expression is

(6) $$\begin{array}{c} g\left(s\right)=\frac{1}{1+e^{-s}}. \end{array}$$

The function *h* is a logistic regression function, and by substituting the function *g*, we can get

(7) $$\begin{array}{c} h_{\vartheta }\left(w\right)=\frac{1}{1+e^{-\vartheta^{T}x}}. \end{array}$$

The function *h* represents the probability that the output is 1 according to *w* when the input feature is *w*. For example, the meaning of *h*_*ϑ*_(*w*) = 0.8 is that the patient has an 80% chance of having a malignant tumor.

The cost function is used to compare the difference between the results predicted by the model and the actual results under a certain parameter. The cost function of logistic regression is

(8) $$\begin{array}{c} J\left(\vartheta \right)=\frac{1}{q}\overset{q}{\underset{i=1}{\sum }}\text{C}\text{ost}\left(h_{\vartheta }\left(\left(w^{\left(i\right)}\right),k^{\left(i\right)}\right)\right). \end{array}$$

Among

(9) $$\begin{array}{c} \text{Cost}\left(h_{\vartheta }\left(w,k\right)\right)=\left\{\begin{array}{cc} -\log\left(h_{\vartheta }\left(w\right)\right), & \text{if }k=1,\\ -\log\left(1-h_{\vartheta }\left(w\right)\right), & \text{if }k=0. \end{array}\right. \end{array}$$

After merging, we can get

(10) $$\begin{array}{c} J\left(\vartheta \right)=-\frac{1}{q}\left[\overset{q}{\underset{i=1}{\sum }}k^{\left(i\right)}\log\left(h_{\vartheta }\left(w^{\left(i\right)}\right)\right)+\left(1-k^{\left(i\right)}\right)\log\left(1-h_{\vartheta }\left(w^{\left(i\right)}\right)\right)\right]. \end{array}$$

The training model finds the parameter *ϑ* that minimizes the loss function *J*(*ϑ*), and the gradient descent method is used in the iterative update. The update rules for parameters are

(11) $$\begin{array}{c} \vartheta_{j}=\vartheta_{j}-\alpha \frac{\partial }{\partial \vartheta_{j}}J\left(\vartheta \right). \end{array}$$

After finding the partial derivative and entering it, the iterative update rule can be obtained as follows:

(12) $$\begin{array}{c} \vartheta_{j}=\vartheta_{j}-\alpha \frac{1}{q}\overset{q}{\underset{i=1}{\sum }}\left(h_{\vartheta }\left(w^{\left(i\right)}\right)-k^{\left(i\right)}\right)w_{j}^{\left(i\right)}. \end{array}$$

#### 3.1.3. Hidden Markov Model

The hidden Markov model (HMM) can use the given observations and assumptions about the working principle to find the hidden state of the system. The key is to determine unknown parameters from known parameters and then analyze and predict [13, 14]. The Markov chain treats the time sequence as a chain, and the value of each node is only related to the *z* nodes in front of it. The sequence generated by the hidden Markov chain is called the state sequence, and the sequence generated by it is called the observation sequence, and the observation sequence is not unique. Supposing *S* = {*s*_1_, *s*_2_, ⋯, *s*_*n*_} is the set of all possible states, *P* = {*p*_1_, *p*_2_, ⋯, *p*_*m*_} is all possible observed states, *L* = {*l*_1_, *l*_2_, ⋯, *l*_*t*_} is the sequence of states, and *Q* = {*q*_1_, *q*_2_, ⋯, *q*_*t*_} is the sequence of observations. Among them, *s* is unknown, and *p* is observable, and the model can be regarded as a quintuple {*S*, *P*, *L*, *Q*, *π*}, corresponding to two states and three matrices:

1. Implicit state *S*: *S* = {*s*_1_, *s*_2_, ⋯, *s*_*n*_}, there are *n* possible states
2. The observable state *P*: *P* = {*p*_1_, *p*_2_, ⋯, *p*_*m*_} has m possible output states
3. State transition matrix *A*:

(13) $$\begin{array}{c} A={\left[a_{ij}\right]}_{n\times n}, \end{array}$$

where

(14) aij=Kit+1=sit=sij, i=1,2,⋯,n, j=1,2,⋯,n,

where *a*_*ij*_ is the state transition probability

(4) Observation probability matrix *B*:

(15) $$\begin{array}{c} B={\left[b_{j}\left(v\right)\right]}_{n\times m}, \end{array}$$

(16) bjv=Kqt=pit=sjv, v=1,2,⋯,m, j=1,2,⋯,n,

where *b*_*j*_(*v*) is the observation probability

(5) Initial state probability vector *π* = {*π*_1_, *π*_2_, ⋯, *π*_*n*_}

Hidden Markov models include the following problems: evaluation, decoding, and prediction. Taking a user visiting a website as an example, the user can register, browse, purchase, or cancel an account. Through the analysis of user behavior to discover potential consumer groups, transition probability records a lot of information about user behavior patterns, through which the relationship between user behavior and time changes can be observed. When a given observation is known, its implicit state is determined by the user's behavior [15]. Evaluation is a probabilistic calculation problem, referring to what is the probability of a sequence occurring given known user state transitions and observations. Decoding is a learning problem, which refers to what is the most likely hidden state of a sequence given it. Prediction refers to finding out what the most likely behavior of the user will be given a sequence of observations.

For information extraction, it mainly solves the decoding and prediction problems. The supervised parameter estimation of the HMM is carried out by the maximum likelihood method, and the unsupervised Baum-Weich algorithm is used for training and learning. After the model parameters are obtained, the Viterbi algorithm is used to decode and output the most likely state label sequence. The specific steps are as follows:

1. First, it is necessary to estimate the parameters of the HMM. Assuming that the number of transitions from state *s*_*i*_ at time *t* to state *s*_*i*_ at time 1 + 1 in the sample is *A*_*ij*_, then the state transition probability *a*_*ij*_ is

(17) $$\begin{array}{c} a_{ij}=\frac{A_{ij}}{\sum_{v=1}^{m}A_{ij}},\;i=1,2,\cdots ,n,\;j=1,2,\cdots ,n. \end{array}$$

Assuming that the number of times the state is *s*_*j*_ at time *t* in the sample is *B*_*jv*_, the observation probability *b*_*j*_(*v*) is

(18) $$\begin{array}{c} b_{j}\left(v\right)=\frac{B_{jv}}{\sum_{v=1}^{m}B_{jv}},\;j=1,2,\cdots ,n,\;v=1,2,\cdots ,m, \end{array}$$

where *s*_*i*_ is the frequency at which the initial state is *s*_*j*_.

(2) After the parameters of the model are obtained, when a sequence *Q* = {*q*_1_, *q*_2_, ⋯, *q*_*t*_} is given, the Viterbi algorithm is used, as shown in Figure 4, to predict the most likely sequence of state labels. The purpose of the Viterbi algorithm is to find the state of each point and make the sequence result optimal. It decomposes the global optimal problem and converts it into the optimal result of each stage

### 3.2. Clinical Features of Gestational Hypertension

The pathogenesis of gestational hypertension is complex, including placental factors, genetic factors and immunity, damage to vascular endothelial cells, nutritional deficiencies, and insulin resistance. Some scholars put forward the “two-stage” theory. The first stage is the preclinical stage, that is, uterine spiral artery trophoblast remodeling disorder, which causes placental implantation, placental ischemia, and hypoxia and releases a variety of placental factors. In the second stage, placental factors enter the maternal blood circulation, promote the activation of systemic inflammatory response and vascular endothelial cell damage, and then cause a series of clinical symptoms such as preeclampsia and eclampsia.

Hypertensive disorders of pregnancy are one of the most common complications in obstetrics, occur after 20 weeks of gestation, and are characterized by hypertension, edema, and proteinuria, along with functional impairment or defects in multiple vital organs of the body, with coma, convulsions, heart failure, placental abruption, disseminated intravascular coagulation, cerebral hemorrhage, and even death. The pathological change of PIH is systemic arterial spasm [16].

#### 3.2.1. Edema

A reasonable weight gain for a normal healthy pregnant woman is 0.5 kg per week. Pregnancy is a physiological phenomenon unique to women, and the normal changes in pregnant women during pregnancy can prevent the return of the inferior vena cava, resulting in fluid retention, which in turn causes edema. If the pregnant woman gained more than 1.0 kg per week, it suggested the possibility of occult edema; when the pregnant woman gained more than 2.0 kg per week, it was regarded as a warning value of potential edema. If there is too much fluid accumulation in pregnant women, pitting edema of the lower extremities can be seen on clinical examination. The occurrence of edema mostly starts at the ankle and gradually develops upward. Both the calf and both feet show pitting edema, and the edema cannot be relieved even if the pregnant woman rests for 6 hours or more and is rated as (+). Edema develops and spreads until the thigh is rated (++), at which point the disease is usually clinically significant. The edema which continued to develop and did not relieve until the vulva, abdomen, and other parts were rated as (+++). Systemic edema was rated as (++++), and pleural effusion may be complicated by this period.

#### 3.2.2. Hypertension

Before the gestational age of pregnant women reaches 20 weeks, their blood pressure is basically the same as before pregnancy or slightly lower. When the gestational age of pregnant women reaches 20 weeks and above, the blood pressure level remains at 140/90 mmHg (1 mmHg = 0.133 kPa), the systolic blood pressure rises more than 30 mmHg, and the diastolic blood pressure rises more than 15 mmHg, it is abnormal.

#### 3.2.3. Urine Protein

Proteinuria usually occurs when pregnant women experience swelling or elevated blood pressure. If proteinuria persists for a long time, pregnant women should be checked for kidney disease. The occurrence of proteinuria indicates a corresponding increase in the permeability of the glomerulus. If the result of routine urinalysis is usually urine protein (+) or the 24 h urine protein quantification is higher than 500 mg, it can be determined as pathological change.

#### 3.2.4. Pathological Changes of Fundus

The pathological changes of the fundus are one of the important indicators to assess the severity of gestational hypertension. The pathological changes of fundus in patients with gestational hypertension can be divided into three stages. The first stage of pathological change is vasospasm. During this period, the diameter of the arterial vessels is not uniform, the reflection effect of the vessel wall is enhanced, and the arterial : venous ratio is 1 : 2 or 1 : 3. The second pathological change is hardening of the blood vessels: during this period, the patient develops edema and sweating. The third stage of pathological changes is the pathological changes of the retina: edema is significant in this stage, and the exudate is flocculent. In severe cases, it can even cause retinal detachment. At this time, the patient's vision will be affected; there is blurred vision and even blindness in severe cases [17]. Most of the above lesions can be recovered after childbirth, and the visual acuity also improves.

#### 3.2.5. Other Clinical Features

Patients with gestational hypertension may also experience dizziness, headache, upper abdominal pain, blind spots, convulsions, nausea, vomiting, and disturbance of consciousness. In severe cases, it may even cause placental abruption, heart failure, and pleural effusion.

## 4. Experiment and Analysis of Adjuvant Therapy with Vitamin E and Astragalus

### 4.1. Clinical Data

#### 4.1.1. Western Medicine Diagnostic Criteria

Gestational hypertension is defined as first-onset hypertension after 20 weeks of gestation, systolic blood pressure ≥ 140 mmHg (1 mmHg to 0133 kPa), and/or diastolic blood pressure 290 mmHg, returning to normal within 12 weeks after delivery. Urine protein tests are negative, and some patients may experience epigastric discomfort or platelet abnormalities. Severe gestational hypertension is defined as systolic blood pressure ≥ 160 mmHg and/or diastolic blood pressure ≥ 110 mmHg [18, 19].

#### 4.1.2. Diagnostic Criteria of Traditional Chinese Medicine

Diagnostic criteria of traditional Chinese medicine include weak blood.

Main symptoms include dizziness after 20 weeks of pregnancy, or edema, aggravated by movement or exertion.

Minor symptoms include palpitations, forgetfulness, less sleep, and more dreams; headache; fatigue, shortness of breath, and lazy words; and pale or chlorotic complexion.

Tongue pulse means pale tongue and thin and weak pulse.

(The above main symptoms must be met, and the secondary symptoms only need to have 1~2 items, plus the tongue and pulse to diagnose the disease.)

#### 4.1.3. Case Selection Criteria

1. Meeting the abovementioned diagnostic criteria for gestational hypertension in Western medicine
2. Meeting the abovementioned diagnostic criteria of traditional Chinese medicine for deficiency of qi and blood
3. Age of 22-38 years
4. Gestational age of 25-33 weeks
5. Systolic blood pressure 140-155 mmHg and (or) diastolic blood pressure 90-105 mmHg
6. No history of hypertension or diabetes before pregnancy, and the biochemical series and routine blood and urine examinations all within the normal range
7. Pregnant women and their families voluntarily participate and sign the informed consent form and take the initiative to receive treatment

### 4.2. Methods

#### 4.2.1. Grouping Method

A total of 120 patients with gestational hypertension who met the inclusion and diagnostic criteria were divided into an experimental group, a vitamin E control group, and a traditional Chinese medicine control group, with 40 cases in each group.

#### 4.2.2. Treatment Methods

*Preparation of astragalus formula granules*: take about 2 kg of astragalus each time and put it into a stainless steel container or pot. Add water for the first time, soak the medicine for about 60 minutes, add water for the second time, continue cooking for about 30 minutes, and mix the two decocting agents. The drug solution was filtered, the residue was filtered, and the paste was concentrated with a relative density of about 1 : 30 (50°C). It is then dried in a vacuum, and the obtained dry extract is powdered and granulated, and the concentration of the ethanol solution is 95%. After drying, 800 grams of granules can be taken each time and placed in the special medicine bag of the hospital; pay attention to drying the medicine.

*Astragalus formula granules*: the dose per bag is about 1.5 g, which is equivalent to 10 g of traditional decoction pieces, 3 bags each time, twice a day, with warm water. Astragalus is shown in Figure 5.

*Commonly used vitamin E tablets*: 50 mg each time, twice a day, taken with warm water. Vitamin E is shown in Figure 6.

*Western medicine routine therapy*: patients with gestational hypertension should try to rest and take a lateral position, strengthen nutrition, and eat more food rich in high protein, iron, calcium, zinc, and other trace elements. Ensure adequate protein and calories, but it is not recommended to limit the intake of salt; intermittent oxygen inhalation (2 L/min); sedation treatment; if necessary, 2.5-5 mg of diazepam can be added before going to bed to ensure adequate sleep.

*Astragalus control group*: on the basis of conventional Western medicine, add astragalus granules orally, 3 bags each time, twice a day, and take with warm water.

*Vitamin E control group*: on the basis of conventional Western medicine, vitamin E tablets were added, 50 mg each time, and the usage was the same as above.

*Experiment group*: on the basis of conventional Western medicine therapy, astragalus granules and vitamin E tablets were added, and the usage and dosage were the same as above.

*Course of treatment*: all three groups of patients were treated until 36 weeks of pregnancy. Before 36 weeks of pregnancy, midwifery check-ups are performed every 2 weeks. After 36 weeks of pregnancy, if there are no special circumstances, then midwifery check-ups can be performed once a week. Pay attention to measure 24 h urine protein, mean arterial pressure, and body mass index, and deliver in hospital, and record the prenatal and postnatal conditions. Instruct patients to avoid cold, spicy, and greasy food when taking the medicine and to live a normal life.

#### 4.2.3. Observation Indicators

Observation indicators include maternal gestational age, gestational week, parity, education level, and body mass index.

1. General physical examination items including body temperature, respiration, and pulse
2. Hematuria series, blood type, coagulation series, and other routine tests
3. ECG, liver and kidney function, biochemical series, and blood sugar examination
4. Ultrasound examination (checking the condition of amniotic fluid and the maturity of the placenta, etc.) and fetal heart rate monitoring

### 4.3. Results

The comparison of the age of onset of the three groups of patients is shown in Table 1, and the comparison of the gestational weeks of the three groups of patients is shown in Table 2. The comparison of parity among the three groups of patients is shown in Table 3. The comparison between the three groups of patients in the disease composition ratio is shown in Table 4.

The results of TCM syndrome efficacy are shown in Figure 7.

The distribution of maternal delivery outcomes and neonatal perinatal outcomes among the three groups is shown in Figure 8.

The comparison of the mean pulsatile pressure and 24 h urine protein data of the three groups of patients before and after treatment is shown in Figure 9.

### 4.4. Result Analysis

1. A total of 120 cases were selected for this clinical trial, ranging in age from 22 to 38 years, with an average age of 30.24 + 2.98 years. The gestational weeks ranged from 25 to 33 weeks, with an average gestational age of 29.00 + 1.92 weeks, with 90 primiparas and 30 multiparous women. The following are the results of comparability analysis of general data: there was no difference in age, gestational age, and parity among the three groups, and the difference was not statistically significant (*P* > 0.05), which was balanced and comparable
2. In comparing the total scores of TCM syndromes in the three groups before treatment, *P* > 0.05, there was no difference in the results, and the difference was not statistically significant, indicating that the overall TCM scores before treatment were balanced. Compared with the total score of TCM syndromes in the three groups after treatment, *P* < 0.05, the results were different, and the difference was statistically significant. The curative effect of the experimental group was better than that of the other two groups. Compared with the total score of TCM syndromes before and after treatment in the experimental group and the astragalus control group, *P* < 0.05, the results are different, and the difference is statistically significant, indicating that both groups can improve the clinical symptoms of the patients, and the therapeutic effect of the experimental group is better than that of the control group astragalus. Compared with the vitamin E control group before and after treatment, *P* > 0.05, there was no difference in the results, and the difference was not statistically significant, indicating that the clinical symptoms were not significantly improved before and after treatment. The author thinks that it is mainly related to the effects of astragalus to invigorate qi and raise yang, strengthen the body and eliminate pathogenic factors, and nourish the heart and dredging the pulse. Secondly, it is believed that vitamin E plays an important role in the normal reproductive process and physiological process and can enhance the body's immunity, and vitamin E can synergistically enhance the function of astragalus, so it can improve the total score of TCM syndromes [20]
3. The degree of urinary protein leakage in the three groups before treatment was compared with *P* > 0.05, there was no difference in the results, and the difference was not statistically significant, indicating that there was no difference in the degree of urinary protein leakage in the three groups before treatment, and the balance was comparable. After treatment, the three groups were compared with those before treatment, all *P* < 0.05, the results were different, and the difference was statistically significant, indicating that the degree of urinary protein leakage in the three groups after treatment was improved, and the experimental group was better than the other two groups. The authors believe that it is mainly related to astragalus dilating blood vessels, diuresis, central nervous system peptide, and renin-angiotensin-aldosterone system to reduce blood pressure. It is closely related to the antioxidant effect of astragalus and vitamin E to improve the damage of vascular endothelium, and from the perspective of traditional Chinese medicine, astragalus also has the effect of diluting water and swelling; thereby reducing the damage to the kidneys, it can effectively improve the degree of leakage of proteinuria
4. Compared with the mode of delivery of the three groups of patients, *P* < 0.05, the results were different, and the difference was statistically significant. Compared with the traditional Chinese medicine control group and the vitamin E control group, the experimental group had more vaginal births, and the cesarean section rate was significantly lower than that of the other two groups. The purpose of hypertensive disease during pregnancy is to control the condition, prolong the gestational age, and ensure the safety of mother and child. The authors believe that astragalus and vitamin E can effectively prevent and treat hypertensive diseases during pregnancy and can expect full-term gestational weeks as much as possible, so it can reduce the proportion of cesarean section to a certain extent [21]
5. The neonatal perinatal outcomes of the three groups of patients were compared *P* < 0.05, the results were different, and the difference was statistically significant. By pairwise comparison of the results, between the experimental group and the traditional Chinese medicine control group, *P* < 0.05, there was a significant difference; the difference was statistically significant; between the experimental group and the vitamin E control group, *P* > 0.05, the difference was not statistically significant. Compared with the vitamin E control group, *P* > 0.05, the difference was not statistically significant. It shows that the effect of the experimental group on neonatal perinatal outcomes is better than that of the traditional Chinese medicine control group and the vitamin E control group. The author believes that astragalus and vitamin E can effectively intervene in gestational hypertension and expect full-term gestational weeks, and the proportion of normal newborns is more
6. Before treatment, the systolic blood pressure and diastolic blood pressure of the three groups were increased to different degrees compared with normal; compared with *P* > 0.05, there was no difference in the results, and the difference was not statistically significant. It indicated that the systolic blood pressure and diastolic blood pressure of the three groups of patients before treatment were comparable. After treatment, the mean arterial pressure was used for a comprehensive comparison. After treatment, the three groups were compared with those before treatment, all *P* < 0.05. The results were different, and the difference was statistically significant, indicating that the blood pressure of the three groups decreased to varying degrees after treatment. The experimental group decreased more significantly than the other two groups. The authors believe that it is mainly related to astragalus dilating blood vessels, diuresis, central nervous system peptide, and renin-angiotensin-aldosterone system to achieve the effect of lowering blood pressure. Astragalus is closely related to the antioxidant effect of vitamin E to improve the damage of vascular endothelium, so it can effectively reduce the mean arterial pressure

## 5. Discussion

First of all, through the study of relevant knowledge points of literature works, this paper initially masters the relevant basic knowledge and analyzes how to conduct research on the risk and clinical treatment of pregnant women during pregnancy based on hypertension. The learning model is expounded, the support vector machine is mainly studied, the clinical characteristics of gestational hypertension are explored, and the clinical therapeutic effect of vitamin E and astragalus in adjuvant treatment of gestational hypertension is analyzed by experiments.

As one of the necessary trace elements in the human body, vitamin E mentioned in this article plays an important role in the normal reproductive process and physiological process. The main trace element contained in astragalus is selenium, and both selenium and vitamin E are antioxidants. Regardless of selenium deficiency or vitamin E in the body, the body's antioxidant capacity will be weakened. However, there is an imbalance between antioxidant and oxidative effects on patients with gestational hypertension, which leads to increased free radical generation and damage to the vascular endothelium [22, 23].

In this paper, the experimental analysis shows that vitamin E plays an important role in the normal reproductive process and physiological process, and astragalus also has the effect of diuretic and swelling; thereby reducing the damage to the kidney, it can effectively improve the degree of proteinuria leakage. Astragalus and vitamin E have a close relationship with the antioxidant effect to improve the damage of vascular endothelium, and both can effectively prevent and treat hypertensive disorders in pregnancy.

## 6. Conclusions

This topic is about the study of hypertensive disorders in pregnancy. Due to the influence and limitation of objective factors such as time and funds, as well as the patient's refusal to accept minimally invasive tests such as laboratory, and the difficulty of case collection, the research sample content is small. There is a certain error in the research results of astragalus combined with vitamin E in the treatment of gestational hypertension. It is necessary to continue to expand the sample content in future clinical trials and research and to conduct long-term efficacy observation and corresponding follow-up of the subjects as much as possible. And in order to further explore its related mechanism of action, corresponding animal experimental studies can be carried out in the later plan. The etiology of hypertensive disorders in pregnancy is complex, and some critical situations may occur at any time during the development of the disease. However, the TCM classification of pregnancy-induced hypertension syndrome is very subjective and simple, and a single rule has not yet been formed [24]. Therefore, traditional Chinese medicine is rarely used in clinical practice to prevent and treat this disease. It is hoped that this clinical trial can provide some reference value for the clinical prevention of the occurrence and development of this disease.

## Figures and Tables

**Figure 1:** Linear classifier.

**Figure 2:** Separating hyperplane.

**Figure 3:** Support vector machine.

**Figure 4:** Viterbi algorithm.

**Figure 5:** Astragalus.

**Figure 6:** Vitamin E.

**Figure 7:** Results of the efficacy of TCM syndromes in the three groups.

**Figure 8:** Distribution of delivery and neonatal perinatal outcomes among the three groups of pregnant women.

**Figure 9:** Comparison of mean pulsatile pressure and 24 h urine protein data before and after treatment in the three groups.

**Table 1:** Age distribution of the three groups ($\bar{x}\pm s$).

Evaluation indicators	Test group	Astragalus control group	Vitamin E control group	*F* statistic	*P*
Age				0.29	0.75^▲^
Mean + SD	31.05 ± 4.59	30.20 ± 3.20	30.90 ± 2.75		
Min–max	22~38	23~35	24~36		
95% CI (*L* ~ *H*)	23.81~33.16	28.61~31.64	29.33~32.33		
*N*	40	40	40		

Note: one-way analysis of variance was used; ▲: compared with the age of the three groups, *P* > 0.05.

**Table 2:** The distribution of gestational age in the three groups ($\bar{x}\pm s$).

Evaluation indicators	Test group	Astragalus control group	Vitamin E control group	*F* statistic	*P*
Gestational week (week)				2.19	0.12^▲^
Mean + SD	29.40 ± 1.80	29.10 ± 2.13	30.75 ± 3.31		
Min–max	26~31	25~32	24~30		
95% CI (*L* ~ *H*)	28.64~30.21	28.18~30.13	27.40~29.18		
*N*	40	40	40		

Note: one-way analysis of variance was used; ▲: comparison of gestational weeks among the three groups, *P* > 0.05.

**Table 3:** Parity distribution of the three groups.

Evaluation indicators	Test group	Astragalus control group	Vitamin E control group	*F* statistic	*P*
Parity (example)				0.53	0.77^▲^
Primipara	28	30	32		
Multiparous	12	10	8		
*N*	40	40	40		

Note: nonparametric test was used for analysis; ▲: comparison of the educational level of the three groups of patients, *P* > 0.05.

**Table 4:** Distribution of the three groups of diseases.

Evaluation indicators	Test group	Astragalus control group	Vitamin E control group	*χ* ^2^ statistic	*P*
Disease composition ratio (cases)				0.44	0.80^▲^
Gestational hypertension	16	14	12		
Mild preeclampsia	24	26	28		
*N*	40	40	40		

Note: row *x* list chi-squared test was used for analysis; ▲: comparison of disease constituent ratios among the three groups of patients, *P* > 0.05.

## Data Availability

No data were used to support this study.
